The article "Technological and antioxidant properties of proteins obtained from waste potato juice" was published in 2020. Journal: Open Life Sci.

# Technological and antioxidant properties of proteins obtained from waste potato juice

**DOI:** 10.1515/biol-2020-0046

**Published:** 2020-06-11

**Authors:** Paweł Jeżowski, Karolina Polcyn, Agnieszka Tomkowiak, Iga Rybicka, Dominika Radzikowska

**Affiliations:** Institute of Chemistry and Technical Electrochemistry, Poznan University of Technology, Poznań, Poland; Students’ Scientific Club of Food Technologists, Poznań University of Life Sciences, Poznań, Poland; Department of Genetics and Plant Breeding, Poznań University of Life Sciences, Poznań, Poland; Department of Technology and Instrumental Analysis, Poznań University of Economics and Business, Poznań, Poland; Department of Agronomy, Poznań University of Life Sciences, Poznań, Poland

**Keywords:** potato juice, by-product, potato juice protein, oil-absorption capacity and water-binding capacity, antioxidative, mineral compounds

## Abstract

The article presents the technological and antioxidant properties of potato juice (PJ) protein concentrate obtained by the novel ultrafiltration method. Commercial products, obtained from waste PJ by the traditional method of acid coagulation of proteins, were studied for comparison. Functional properties such as water or oil absorption, foaming capacity, and foam stability (FS) as well as solubility at various pH were assessed. Moreover, the total phenolic compound content, antioxidant activity, and mineral composition were determined. The results showed that PJ protein concentrate obtained by ultrafiltration has good oil absorption properties (6.30 mL/g), which is more than two times higher than the commercial proteins used in the comparison (P2 = 2.33 mL/g and P3 = 2.67 mL/g). Moreover, the ability to create and stabilize foam was also higher (FS ranging from 20.0% at pH = 10 to 11.3% at pH = 2 after 60 min of testing). It had higher content of macro- and microelements and antioxidant activity compared to other samples. Therefore, it is possible to obtain interesting potato protein concentrate from the waste product of the starch production process, which may be an interesting raw material for enriching food.

## 1 Introduction

Factories processing raw plant materials produce a number of by-products and waste products that pose a problem related to their disposal. At the same time, they can be a potential source of ingredients that could be used in food production. Starch has been used in the production of food [1,2] for a long time, but it also has other applications [3,4]. Potato juice (PJ) is one of the more interesting by-products of starch production [5,6]. Fresh PJ contains approximately 1% of mineral compounds and 4% of organic compounds, mainly protein (2%) [7]. In addition, PJ is rich in biologically active compounds such as β-carotene, polyphenols, ascorbic acid, tocopherol, or α-lipoic acid [8,9]. Published studies show that PJ is an interesting raw material in food production due to its biological activity. PJ was used in folk medicine for a long time to treat many gastrointestinal diseases [10,11]. However, the scientific research about its safety and effectiveness as a treatment substance began only in the twenty-first century. Kujawska et al. [12] reported the anti-inflammatory effect of PJ. Until now, PJ has not been used in human nutrition, mainly due to the content of antinutritional substances – glycoalkaloids (solanine and chaconine) [13]. Despite the fact that technologies for the production of valuable metabolites by microbiological methods using PJ [14,15,16] or health-promoting food products containing PJ have been developed [17,18,19,20,21], currently the main technique for managing of PJ is the production of potato protein concentrates by the acid-thermal coagulation, and used as animal feed [22].

The article "Technological and antioxidant properties of proteins obtained from waste potato juice" was published in 2020. Journal: Open Life Sci.

Protein preparations used as food ingredients should have a favorable chemical composition and high nutritional value. One of the important aspects is the functional properties responsible for creating the right structure of food enriched with protein and consequently obtain a product with the desired sensory characteristics [23,24]. For many authors, the functional properties of proteins are the key criteria for their possible use as food ingredients. However, the origin of the protein and the various methods used to isolate it can limit the precise determination of their functional properties. The main functional properties of proteins include water absorption, oil absorption, foam formation, and stabilization as well as solubility at various pH [25,26]. Protein preparations with appropriate functional properties can favorably affect the characteristics of food products, giving them the desired color, texture, and aroma.

The solubility of protein preparations affects their biological value, structure-forming capacity, and enzymatic activity [27,28]. Proteins with a relatively high electric charge and low hydrophobicity usually dissolve easily in water, while proteins with a high content of hydrophobic amino acid residues are soluble in the organic solvents [29]. Protein solubility depends on the method of preparation, temperature, protein concentration, and ionic strength [30,31]. Water absorption of proteins is defined as the ability to bind and retain water in a physicochemical or physical way, regardless of heating or gravity. It is a critical factor in assessing the functional properties of proteins because it affects the sensory properties of food products. Oil absorption of proteins, i.e., their ability to retain and absorb fat, consists in the physical entrapment of fat globules [32,33]. It basically affects the texture as well as other quality characteristics of finished products. Proteins that are not soluble in water and salt solutions as well as hydrophobic proteins are characterized by good fat-binding capacity. Oil absorption is important to emphasize the taste and appearance of food products [34]. Foam formation is determined on the basis of foam volume increase due to whipping and is expressed most often in percentage [26]. Protein solutions achieve the greatest frothiness within the isoelectric point. The ability to create foams is of great importance in the formation of desirable sensory features, e.g., texture of confectionery, bread, or whipped cream [35,36,37,38]. Foam stability (FS) expresses the ability to maintain the maximum volume over a specified period of time, and this property is very desirable in the production of confectionery. FS is responsible for the developed polypeptide chains accumulating at the water/air interface.

The article "Technological and antioxidant properties of proteins obtained from waste potato juice" was published in 2020. Journal: Open Life Sci.

The aim of this work was to analyze the functional properties of PJ protein concentrate obtained by the novel ultrafiltration method. Basic features determining the technological usefulness of the protein, i.e., water absorption, oil absorption, and ability to form foam and its stabilization as well as solubility at various pH, were analyzed.

## 2 Materials and methods

### 2.1 Materials

The first potato protein was obtained from waste PJ (PPZ “Trzemeszno”, Poland) by ultrafiltration in accordance with the method previously described by Kowalczewski et al. [39], denoted in the text as P1. Briefly, the experiment was carried out in an open system in which the permeate was discharged into a separate container (concentration mode). Concentration was performed at a transmembrane pressure of 400 ± 15 kPa, a cross-flow velocity inside the membrane of 0.5 ms^−1^, and a temperature of 20°C. The obtained content was further directed to the spray-drying process to ensure long-term storage stability in a Mobile Minor™ 2000 Spray Dryer (GEA Co., Søborg, Denmark) using the following conditions: 170°C at the inlet to the drying chamber and 95°C at the outlet.

Moreover, two commercial protein concentrates, obtained from PJ by the traditional method of acid coagulation of proteins, were used for comparison: from Royal Avebe U.A., the Netherlands (Solanic^®^100; denoted as P2) and from PPZ Trzemeszno, Poland (denoted as P3).

### 2.2 Basic chemical characteristic

The total nitrogen content in the tested samples was determined by the Kjeldahl method according to ISO 1871 [40]. The total protein content was calculated by multiplying the percentage of nitrogen content by a factor of 6.25. The ash content was determined in accordance with ISO 763 [41]. The moisture content was made in accordance with AACCI 44-19.01 [42]. The concentrations of minerals (Ca, Cu, Fe, K, Mg, Mn, Na, and Zn) were determined using the flame atomic absorption spectroscopy (SpectrAA-800; Varian, Palo Alto, CA, USA) preceded by mineralization with nitric acid [43]. The percentage of population reference intake (PRI) and adequate intakes (AIs) was calculated according to the latest european food safety authority (EFSA) recommendations [44]. The mineral contents were expressed in g/100 g of the sample.

The article "Technological and antioxidant properties of proteins obtained from waste potato juice" was published in 2020. Journal: Open Life Sci.

### 2.3 Antioxidant activity measurements

The extracts of polyphenols were prepared from freeze-dried samples according to the methods described by Miedzianka et al. [45], using 70% aqueous acetone (0.1% acetic acid). One gram of the sample was added to the solvent in a tube, then the mixture was homogenized using a vortex for 30 s, transferred to an ultrasound bath for 5 min, and centrifuged at 10,000 × g for 10 min at 4°C. The extracts were prepared three times, the supernatants were mixed together, and then acetone was evaporated and the remaining aqueous extract was collected.

### 2.4 Determination of total phenolic compounds (TPCs)

The TPC content was determined by the standard Folin–Ciocalteu colorimetric method [46]. Absorbance was measured at 765 nm. The total content of phenolics was expressed in milligrams of gallic acid per gram of product.

### 2.5 Free radical scavenging activity using 2,2′-azinobis[3-ethylbenzthiazoline]-6-sulfonic acid (ABTS)

The ABTS radical cation decolorization assay was determined by the method of Re et al. [47] with slight modifications. The ABTS was dissolved in distilled water to a 7 mM concentration and potassium persulfate was added to achieve a concentration of 2.45 mM. The reaction mixture was left at room temperature overnight (12–16 h) in the dark before use and then diluted with 0.01 M phosphate-buffered saline (pH 7.00) to give an absorbance value of ∼0.70 at 734 nm. The working ABTS solution of 2 mL was mixed with 0.98 mL of PBS and 0.02 mL of sample extract. The absorbance was measured spectrophotometrically 6 min after the addition of the sample. Trolox was used as the standard, and the results were expressed in milligram/gram of Trolox equivalents (Trolox equivalent antioxidant capacity [TEAC]).

### 2.6 Effect of pH on foaming capacity (FC) and FS

FC and FS were measured according to the method of Waniska and Kinsella [48], with some modifications. One gram of the preparation was weighed into the tube and 200 mL of distilled water was added to it. The resulting mixture was adjusted to the appropriate pH (2, 4, 6, 8, 10, and 12) using 0.5 M NaOH or 0.5 HCl. The sample was then homogenized for 2 min at 16,000 rpm (T10 basic ULTRA-TURRAX^®^; IKA Werke, Germany). The beaten sample was immediately transferred to a measuring cylinder where the total foam volume was determined after 0, 5, 10, 30, and 60 min. FC and FS were calculated according to the following equations:

\text{FC}=(A/B)\times 100,

where *A* denotes the volume after whipping (cm^3^) and *B* is the volume before whipping (cm^3^).

\text{FS}=(C/B)\times 100,

where *B* denotes the volume before whipping (cm^3^) and *C* is the volume after a certain time (cm^3^).

The article "Technological and antioxidant properties of proteins obtained from waste potato juice" was published in 2020. Journal: Open Life Sci.

### 2.7 Water-binding capacity

The method of Timilsena et al. [49] was used for the determination of water-binding capacity. A sample of approximately 1 g was weighed into a test tube and 20 mL of distilled water was added to it. The resulting mixture was shaken using a laboratory shaker. After 15 min, the solution was shaken again for 60 s. Then the precipitate was separated from the supernatant using a centrifuge (4,500 g, 15 min; Rotofix 32A; Merazet, Poland). The separated solid was oven-dried. Water absorption was expressed as the amount of water (g) absorbed by 1 g of the preparation.

### 2.8 Oil-absorption capacity

The oil-absorption capacity was determined using the method of Wu et al. [50]. Briefly, 1 g of preparation was weighed in the test tube and 15 mL of rapeseed oil was added. The whole was shaken using a laboratory shaker. After 30 min, the resulting mixture was separated using a centrifuge (4,000 g, 10 min; Rotofix 32A). Oil absorption was expressed as the amount of oil (milliliter) absorbed by 1 g of the preparation.

### 2.9 Effect of pH on protein solubility

The solubility of protein was determined per the method of Achouri et al. [51] with slight modifications. For determining protein solubility at different pH, 200 mg of preparation was weighed in the tube and 15 mL of distilled water was added and then the pH adjusted (2, 4, 6, 8, 10, or 12) using either 0.5 M NaOH or 0.5 M HCl. The sample was then shaken at room temperature for 30 min and successively centrifuged at 4,500 g for 15 min.

### 2.10 Statistical analysis

All measurements were repeated five times. One-way analysis of variance was performed independently for each variable. Tukey’s honestly significant difference *post hoc* test was used to identify statistically homogeneous subsets at *α* = 0.05. Statistical analysis was performed using Statistica 13 software (Dell Software Inc., Round Rock, TX, USA).

The article "Technological and antioxidant properties of proteins obtained from waste potato juice" was published in 2020. Journal: Open Life Sci.

## 3 Results and discussion

### 3.1 Basic chemical characteristics

The average dry matter, protein, and ash content are given in Table 1. All analyzed samples had similar dry matter content. Its highest share was obtained in P2 (93.61%) but slightly lower in P1 (92.73%) and the lowest in P3 (91.98%).

**Table 1:** Basic chemical characteristics

Sample	Dry matter, %	Protein content,% d.m.	Ash content,% d.m.
P1	92.73 ± 0.27^a^	72.05 ± 0.15^c^	7.29 ± 0.29^a^
P2	93.61 ± 0.15^a^	79.36 ± 0.28^b^	5.72 ± 0.09^b^
P3	91.98 ± 0.05^b^	83.33 ± 0.86^a^	2.20 ± 0.07^c^

Different superscript letters in columns indicate statistically different mean values (*p* < 0.05); d.m. – dry matter.

Table 2 shows the mineral composition of the analyzed samples. The P1 was characterized by high content (in relation to PRI/AI) of most minerals under study, especially K, Mg, Cu, Fe, Mn, and Zn. For example, its 100 g portion realized up to 75% and 169% of daily recommendations of Mg and Fe, respectively. Such high mineral contents make P1 an attractive food additive with a wide spectrum of potential applications in different food matrices, e.g., in the formulation of gluten-free bakery products that are often poor in proteins or minerals [52]. Moreover, the elemental profile of P1 was much more preferable than those of commercial P2 and P3. P1 had a higher content of macro- and microelements compared to other samples. The highest contents were noticed for Ca (almost 3× higher than P2 and 2× higher than P3), Mg (almost 6 and 10 times higher than P2 and P3, respectively), Fe (more than 3 and 6 times higher than P2 and P3, respectively), Mn (6 and 379 times higher than P2 and P3, respectively), and Zn (3 and 86 times higher than P2 and P3, respectively). P1 had a lower content of Na and Cu minerals compared to the commercial PJs. P1 had the lowest Na content among the analyzed samples, but all samples were at the comparable level of 85–129 mg/100 g. P1 contained 1.14 mg of Cu in 100 g, while P2 and P3 possessed 0.48  and 3.40 mg, respectively.

**Table 2:** Results of mineral composition analysis

Mineral	P1		P2		P3	
	mg/100 g	% PRI/AI	mg/100 g	% PRI/AI	mg/100 g	% PRI/AI
Ca	118 ± 8^a^	12	34.0 ± 1.4^c^	3	59.0 ± 0.9^b^	6
K	4,341 ± 271^a^	92	1,021 ± 50^c^	22	3,536 ± 57^b^	75
Mg	241 ± 9^a^	75	41.5 ± 0.9^b^	13	2.3 ± 1.8^c^	0.7
Na	84.5 ± 4.9^c^	6	93.0 ± 4.0^b^	6	129 ± 3^a^	9
Cu	1.14 ± 0.07^b^	127	0.48 ± 0.03^c^	53	3.40 ± 0.01^a^	376
Fe	30.5 ± 4.2^a^	169	12.8 ± 0.6^b^	75	4.6 ± 0.1^c^	26
Mn	3.79 ± 0.17^a^	211	0.56 ± 0.02^b^	6	0.01 ± 0.01^c^	0.8
Zn	6.04 ± 0.11^a^	76	1.8 ± 0.1^b^	22	0.07 ± 0.01^c^	0.9

Different superscript letters in rows indicate statistically different mean values (*p* < 0.05).

The article "Technological and antioxidant properties of proteins obtained from waste potato juice" was published in 2020. Journal: Open Life Sci.

### 3.2 Antioxidant activity

Plants are the source of many bioactive compounds with broad antioxidant, antimicrobial, anti-inflammatory, or even anticancer activity [53,54,55,56,57]. Among the antioxidant substances, phenols are characterized by their highest antioxidant activities [58,59,60]. The published literature data point to the anti-inflammatory effects of potatoes and attribute them to the presence of antioxidants, including phenolic acids, carotenoids, or anthocyanins. The systemic anti-inflammatory effect of potato was confirmed in human cohort studies and correlated with the concentration of some potato antioxidants in blood serum [8,61,62]. The results of the analyses (Table 3) indicate that the potato protein from PJ obtained by the novel method (P1) was characterized by the highest antioxidant activity among all the protein concentrates analyzed, which is consistent with the literature data [39]. It is worth noting that the antioxidant activity of P1 is 15× higher than that of fresh PJ [63]. The highest content in P1 was also observed for the total content of polyphenolic compounds. The high content of polyphenolic compounds, higher than that in flesh-colored potatoes that are rich in anthocyanin pigments and polyphenols [64], indicates that the potato protein concentrate not only can be used as an additive in bioactive food but also reduces fat oxidation [65].

**Table 3:** Antioxidant activity expressed as the TEAC and TPC contents

Sample	TEAC, mmol/g	TPC, mg/g
P1	1.61 ± 0.16^a^	2.21 ± 0.21^a^
P2	1.26 ± 0.19^b^	2.02 ± 0.11^a^
P3	0.91 ± 0.24^b^	1.43 ± 0.18^b^

Different superscript letters in columns indicate statistically different mean values (*p* < 0.05).

### 3.3 Oil-absorption and water-binding capacity

The usefulness of protein preparations as food ingredients is based on their technological properties, which closely refer to the physicochemical properties that affect the processing and behavior of proteins in food products. The main functional properties of proteins are solubility, FC, FS, water-binding capacity, and oil-absorption capacity.

Good water absorption by the protein preparations depends on several parameters such as the appropriate amount of hydrophilic groups, methods of protein precipitation, and environmental reaction [66,67,68]. The data in Table 4 show that both P2 (3.68 mL/g) and P3 (3.37 mL/g) had better water absorption than P1 (1.69 mL/g). This is probably due to the fact that P1 has a high solubility (Figure 2), while carbohydrate residues and constituents of other protein concentrates may improve water binding. The differences may also indicate that the total protein content and changes in their structure are due to the conditions of their isolation [69]. Another study about PJ protein isolates shows water absorption results at the level of 2.73 g/g [70]. Piecyk and Klepacka [71] presented that heating of protein preparations obtained from bean seeds resulted in a significant improvement in water absorption. The greater capacity of water binding in protein preparations makes them more suitable additives where hydration is required, as is the case of bread and cake.

The article "Technological and antioxidant properties of proteins obtained from waste potato juice" was published in 2020. Journal: Open Life Sci.

**Table 4:** Comparison of oil-absorption and water-binding capacities

Sample	Water absorption, mL/g	Oil absorption, mL/g
P1	1.69 ± 0.18^c^	6.30 ± 1.56^a^
P2	3.68 ± 0.10^a^	2.33 ± 0.31^b^
P3	3.37 ± 0.19^b^	2.67 ± 0.76^b^

Different superscript letters in columns indicate statistically different mean values (*p* < 0.05).

**Figure 1:** The results of FC analysis.

The P1 was characterized by a very good oil-absorption capacity. One gram of this preparation absorbed 6.30 mL of oil, which gave more than a twofold higher result compared to the other two analyzed proteins (Table 4). Oil absorption is one of the most important technological properties of protein preparations, as it has a large impact on their activity during the creation and stabilization of emulsions. Protein preparations distinguished by good oil absorption could be used in the production of meat products, meat replacement products as well as fillers for pancakes or soups [66,72]. The mechanism of fat absorption has been explained in the literature as the physical entrapment of oil, and several authors have linked oil-absorption capacity to nonpolar protein side chains as well as to various conformational features of proteins [73,74].

### 3.4 FC and FS

The study showed that P1 has significantly better foaming properties compared to P2 and P3 (Figure 1). P1 shows several times higher FC, with the ability to form foam closely correlated with the pH of the environment. The highest values of 27.5% were observed at pH 4 and 10, and the lowest of 20% and 22.5% were found at pH 2 and 12, respectively. Many authors report that the low FC of protein preparations may be associated with low solubility and surface hydrophobicity of proteins [64,72,75]. Partsia and Kiosseoglou [76] believed that the ability of proteins to form foams is related to their molecular weight and the appropriate amount of exposed active hydrophilic groups. The lower the molecular weight of proteins in the formulation, the better the foaming activity. Lighter particles more easily penetrate and remain on the interface. PJ consists of soluble and insoluble protein fractions. Insoluble fractions constitute about 25% of proteins and in crystalline form in cell juice. However, the soluble fractions of potato proteins constitute about 75–80%, and they consist mainly of globular proteins (50–60% albumin, 25–16% globulin, 2–4% prolamin, 9% gluten, and 9% the so-called residual proteins). The mixture of albumin and globulins forms a basic group of soluble globular proteins, called tuberine (patatin), with a molecular mass of 44 kDa [77]. Proteins with high FC are desirable in many food applications and are particularly used in aeration and whipping food systems.

The article "Technological and antioxidant properties of proteins obtained from waste potato juice" was published in 2020. Journal: Open Life Sci.

**Figure 2:** Dependence of solubility protein at different pH.

As for the FC, P1 had the best foam stabilization properties. Compared to other tested proteins, it showed several times higher stability of the obtained foam at each of the analyzed pH (Table 5). The optimal conditions for the foam formation were at pH 10. However, as time progressed, foam durability decreased. Shchekoldina and Aider [78] in their research on the foaming properties of soy and sunflower proteins observed that as the pH increases, the FC and FS increase. The low FC and FS of proteins isolated at acidic pH may indicate insufficient electrostatic repulsion and thus excessive protein–protein interactions in the form of aggregates that are harmful to foam formation. An increase in foam expansion may be due to the increased solubility, rapid development of the air–water interface, limited intermolecular cohesion, and flexibility of protein surfactant molecules.

**Table 5:** Results of the FS analysis of proteins

pH	FS (%)											
	P1				P2				P3			
	5 min	10 min	30 min	60 min	5 min	10 min	30 min	60 min	5 min	10 min	30 min	60 min
2	20.0	17.5	17.5	11.3	—	—	—	—	3.8	3.8	3.0	2.5
4	25.0	23.1	21.9	18.8	—	—	—	—	5.5	5.3	2.0	1.3
6	25.0	20.6	15.9	12.5	5.0	5.0	4.0	3.0	10.0	10.0	7.5	7.5
8	20.0	15.0	13.8	12.5	6.3	6.3	6.3	6.3	5.8	5.8	5.5	5.5
10	27.5	27.5	22.5	20.0	6.3	6.3	6.3	6.3	10.0	6.3	6.3	6.3
12	22.5	22.5	20.0	17.5	11.3	10.0	8.8	8.8	12.5	12.5	12.5	12.5

### 3.5 Protein solubility

Proteins analyzed during the tests showed very low solubility in aqueous solutions (0.001–0.41%; Figure 2). However, after comparing the obtained results, it can be stated that P1 has much better solubility than P2 or P3. P1 obtained the highest solubility of proteins at pH 10 (0.41%) and the lowest at pH 4 (0.15%). Low solubility of proteins could be caused by the denaturing changes [79,80] and reduced interaction between proteins and water, increasing protein–protein interactions, causing their aggregation and precipitation, and hence reducing their solubility. It is believed that increased ionic strength also contributes to the reduction in protein solubility [81]. Holm and Eriksen [82] showed in their research that natural potato protein has better solubility compared to commercial soy protein. While Partsia and Kiosseoglou [76] observed the good solubility of a potato protein preparation obtained with carboxymethyl cellulose in a neutral environment.

The article "Technological and antioxidant properties of proteins obtained from waste potato juice" was published in 2020. Journal: Open Life Sci.

## 4 Conclusion

Based on presented studies, PJ can become a raw material for obtaining protein preparations. The protein concentrate of PJ obtained with the ultrafiltration method has favorable functional properties, including good oil absorption 6.30 mL/g, which is more than two times higher than the commercial proteins used in the comparison (P2 = 2.33 mL/g and P3 = 2.67 mL/g). It showed much better FS ranging from 20.0% at pH = 10 to 11.3% at pH = 2 after 60 min of testing. For comparative reasons, potato proteins available in the market had a lower FS with a maximal value of 12.5% and the lowest one at 1.3% of the analyzed pH. During the tests, the analyzed proteins showed very low solubility; however, after comparing the obtained results, the new PJ protein concentrate solubility was the highest and ranged from 0.15% at pH = 4 to 0.41% at pH = 10, while the solubility of other analyzed proteins reached a maximal solubility of only 0.06% at pH = 12.
